# Diagnosis of Cervical Cancer based on Ensemble Deep Learning Network using Colposcopy Images

**DOI:** 10.1155/2021/5584004

**Published:** 2021-05-04

**Authors:** Venkatesan Chandran, M. G. Sumithra, Alagar Karthick, Tony George, M. Deivakani, Balan Elakkiya, Umashankar Subramaniam, S. Manoharan

**Affiliations:** ^1^Department of Electronics and Communication Engineering, KPR Institute of Engineering and Technology, Avinashi road, Coimbatore, 641407 Tamilnadu, India; ^2^Renewable Energy Lab, Department of Electrical and Electronics Engineering, KPR Institute of Engineering and Technology, Avinashi road, Coimbatore, 641407 Tamilnadu, India; ^3^Department of Electrical and Electronics Engineering, Adi Shankara Institute of Engineering and Technology Mattoor, Kalady, Kerala 683574, India; ^4^Department of Electronics and Communication Engineering, PSNA College of Engineering and Technology, Dindigul, 624622 Tamilnadu, India; ^5^Department of Electronics and Communication Engineering, Vel Tech High Tech Dr. Rangarajan Dr. Sakunthala Engineering College, Tamilnadu 600062, India; ^6^Department of Communications and Networks, Renewable Energy Lab, College of Engineering, Prince, Sultan University, Riyadh 12435, Saudi Arabia; ^7^Department of Computer Science, School of Informatics and Electrical Engineering, Institute of Technology, Ambo University, Ambo, Post Box No. 19, Ethiopia

## Abstract

Traditional screening of cervical cancer type classification majorly depends on the pathologist's experience, which also has less accuracy. Colposcopy is a critical component of cervical cancer prevention. In conjunction with precancer screening and treatment, colposcopy has played an essential role in lowering the incidence and mortality from cervical cancer over the last 50 years. However, due to the increase in workload, vision screening causes misdiagnosis and low diagnostic efficiency. Medical image processing using the convolutional neural network (CNN) model shows its superiority for the classification of cervical cancer type in the field of deep learning. This paper proposes two deep learning CNN architectures to detect cervical cancer using the colposcopy images; one is the VGG19 (TL) model, and the other is CYENET. In the CNN architecture, VGG19 is adopted as a transfer learning for the studies. A new model is developed and termed as the Colposcopy Ensemble Network (CYENET) to classify cervical cancers from colposcopy images automatically. The accuracy, specificity, and sensitivity are estimated for the developed model. The classification accuracy for VGG19 was 73.3%. Relatively satisfied results are obtained for VGG19 (TL). From the kappa score of the VGG19 model, we can interpret that it comes under the category of moderate classification. The experimental results show that the proposed CYENET exhibited high sensitivity, specificity, and kappa scores of 92.4%, 96.2%, and 88%, respectively. The classification accuracy of the CYENET model is improved as 92.3%, which is 19% higher than the VGG19 (TL) model.

## 1. Introduction

Cervical cancer is the second most deadly condition for women in the medical world following breast cancer and later believed that cervical cancer remains incurable in the later stages. Much recent progress has been made to improve the disease detection rate by using an image. Statistics by the World Health Organization (WHO) revealed that cervical cancer is the fourth most prevalent cancer globally, with a reporting rate of 5,70,000 new cases in 2018, accounting for 7.5% of all women cancer deaths [1]. Over 3,11,000 cervical cancer deaths per year were reported at around 85% in low- and intermediate-income countries, and the early diagnosis of cervical cancer offers a way of saving a life. Women with HIV are sixfold more likely to develop cervical cancer than women without HIV, and it is estimated that 5% of all cervical cancer cases are related to HIV. A variety of considerations have redefined screening effectiveness, which includes the access to equipment, consistency of screening tests, adequate supervision, and detection and treatment of lesions detected [2]. Despite severe medical and science advancements, this disease is not completely curable, mainly if diagnosed in a developing state. Prevention and screening services, therefore, play a crucial role in the fight against cervical cancer. The screening of cervical cancer follows a typical workflow: HPV testing, cytology or PAP smear testing, colposcopy, and biopsy. Several tools supported the workflow which have been created to make it more effective, practical, and inexpensive. The PAP smear image screening is mostly employed for the treatment of cervical cancer, but it requires a greater number of microscopic examinations to diagnosis of cancer and noncancer patients, and also it is time consuming and requires trained professionals, but there is a chance of missing the positive cases by using the conventional screening method. The PAP smear and HPV testing are very costly treatment, and it also provides lower sensitivity. On the other side, the colposcopy treatment is widely used in the developing countries. To overcome the shortcomings in PAP smear images and HPV testing, the colposcopy screening is used. Both cervical and other cancers are more likely to be treated in the early stage, but the lack of signs and symptoms at this stage hinders the early diagnosis. Cervical cancer deaths can be avoided by successful screening schemes and can lead to lowered sickness and impermanence [3]. In low- and middle-income nations, cervical cancer screening facilities are very sparse because of a shortage of qualified and educated health care staff and insufficient healthcare funding to fund screening systems [4].

Colposcopy is a popular surgical procedure to prevent cervical cancer. Timely identification and classification of this type of cancer may significantly improve the patient's eventual clinical care. Several works have been taken various approaches for collecting details from images in digital colposcopy. These studies' key aim is to provide health practitioners with tools during colposcopy exams irrespective of their level of competence. Previous studies have been developed in diagnosis using computer-aided systems for a range of tasks, including improvement and evaluation of image quality, regional segmentation, picture identification, identification of unstable regions and patterns, transition zone type classification (TZ) type, and cancer risk classification [5]. CAD instruments help improve the picture of cervical colposcopy and areas of concern segments and identify certain anomalies. These methods help clinicians to make diagnostic choices, but they should have adequate experience and expertise to make an appropriate diagnosis. The appearance of pathological regions may indicate such neoplasms; so in a colposcopy analysis, the detection of these lesions may be very critical. These abnormal areas include acetowhite, abnormal vascularization, mosaic areas, and punctures [6, 7]. Most literature surveys recommended a mechanism to spot irregular areas in conventional colposcopy images. Most works include inconsistent zone segmentation, including exclusion from specular reflection, segmentation of the cervix, acetowhite field segmentation [8], mosaic regions recognition, vasculature and puncture, and classification [9].

Deep learning has made significant advances in different applications such as computer vision, natural language processing, forecasting, and battery health monitoring [10]. Medical image processing, including classification, identification, segmentation, and registration, plays an essential role in disease diagnosis. Medical images such as MRI, CT, and ultrasound images and blood smear images [11], make up the vast majority of the image data processed. Deep learning's multilayer neural network perception mechanism can learn more abstract features in images and is expected to address the issues that plague conventional medical CAD systems. However, the deep learning techniques should be supported with an extensive database, especially for positive cases. To overcome this issue, many transfer learning and ensemble learning approaches are discussed in the previous work. The convolution neural network (CNN) is used to identify MI signals in an efficient computer-aided diagnosis (CAD) framework for urban healthcare in smart cities [12]. The novel feature extraction protocol followed by the genetic algorithm is proposed to detect arrhythmia to improve the performance using several tiers [13]. The structure is as follows: Section 2 discusses the related work connected with cervical screening, Section 3 elaborates the proposed architecture of CYENET to cervical screening, Section 4 interprets the results obtained out of the implementation, and Section 5 drawn the conclusion and future scope of this work.

## 2. Related Work

Several algorithms were utilized for machine learning, and their segmentation refining was matched to a cervical cancer classifier in which random forests showed the best output [14]. Also, robust refinement methods have been used to manage, and unattended learning approaches to the different image or superpixel patches from extracted objects methods include Adaboost detectors [15], SVM supports [16], or Gaussian mixture models [17]. A novel Markov random field segmentation based on superpixels was proposed and implemented for nonoverlapping cells [18]. The multifilter SVM is executed, and the parameters were set for the identification of cervical cells [19]. It was suggested that cervical cell classification using artificial neural networks (ANN) was built and tested with a precision of 78% [20]. Unbalanced medical evidence for the variety of cervical cancer without any parameter change was addressed using an unsupervised approach [21]. The particle swarm optimization (PSO) with KNN membership values outperformed all other fundamental classification models [22]. The cervical cancer cell is classified using shape and texture characteristics of the segmentation and classification method and Gabor characteristics. It was found that a greater accuracy of 89% was obtained for both normal and cancer cell classification [23]. The extracted features from CNN were classified using the least square support vector machine (LSSVM) and produced more remarkable results, one of the suggested model's reference components [24]. Radial basis function- (RBF-) SVM also obtained a strong outcome and outperformed logistic regression and random forest methods [25]. Based on the features, it was found that the accuracies were ranged from 90 to 95%.

New deep architectures such as ResNet, Inception, and tree models [26] have recently shown promising results in many applications and detect cancer cells. As one of the deep learning methods, the convolutional neural networks is the commonly used technique to identify and recognize cervical cancer [27]. Early cervical cancer cell identification and classification method based on CNN's was developed to extract deep learned features from the cervical images [28]. The extreme learning machine (ELM) was used to categorize the input images. The CNN paradigm was used for fine-tuning and transfer learning. Alternatives to classifiers based on the ELM, the multilayered perceptron (MLP), and the automotive encoder (AE) were also studied. It was reported that the stacked soft-max autoencoder reported a 97.25% precision on the cervical cancer dataset [29]. It was concluded that a tentative effort was made to tackle the issue of patient risk prediction using the applications for machine learning to grow cervical cancer. The machine learning software with cervical screening was used to tackle the problem of predicting the patient's risk [30]. They concentrated on the transition of information between linear classifiers to related activities to predict the patient's risk. Since the related risk factors in the population are highly sparsely influenced, the techniques for reducing dimensionality can boost the power of predictive machine learning models [31]. However, several projects benefit from reducing dimensionality and classification by using suboptimal methods in which each part is learned separately [32]. For the efficient collection and classification of cell properties in cervical smeared images [33], a quantum hybrid- (QH-) innovative approach was combined with adaptive search capability of the quantum-behaved particle swarm optimization (QPSO) method with the intuitionist reasonableness of the standard fuzzy *k*-nearest neighboring (fuzzy k-NN) algorithm (known simply as *Q*-fuzzy approach).

A model was suggested for the cervical cancer prediction model (CCPM) that produces an early prediction of cervical cancer with input risk factors [34]. CCPM eliminates outliers first by employing outlier identification methods such as Density-Based Spatial Noise Cluster (DBSCAN) and isolation Forest (iForest) by balancing the number of cases in the dataset. This approach has shown greater accuracy in cervical cancer forecasting. To design an integrated cervical cell diagnostic and screening device, the authors have developed a new Regionally Growing Extraction Function (RGBFE) to extract diagnostic features from the images [35]. Data from the cervical cell images with extracted features were supplied into the intelligent diagnostic component. Precancerous phases were forecasted using a new architecture called the Hybrid Multilayered Perceptron (H2MLP) network using an artificial neural network is created. The cells are classified into normal, low-quality intraepithelesis (LSIL), and high-quality intraepithelesis (HSIL). Improved screening systems are also inaccessible in developing countries, owing to the difficulty and time-consuming nature of manually screening irregular cells from a cervical cytology specimen. This system focused on transfer learning, and pretrained and densely connected convolutional networks are used to suggest a computer-aided diagnostic (CAD) method for automated cervical image classification to assess CIN2 or higher level lesions in the cervical imaging (ImageNet and Kaggle). The effect of various training strategies on model results, including scratch random initialization (RI), pretrained model (FT) tuning, different size of training data, and *K*-fold cross validation, was evaluated. Experimental findings demonstrated accuracy of 73.08% for 600 test images [36]. The summary of the literature related to the screening of cervical cancer is provided in Table 1. Owing to the millions of cells that a pathologist must examine, Pap smear screening takes longer days for analyses. Deep learning models were used to identify all cells and other materials present in the Pap smear image screening. The system is often difficult to classify since two cells overlap. To address the need for this problem, meticulously annotated data is required; developing this form of the medical field dataset is very difficult. Considering the challenges mentioned above, a novel deep learning model for cervical cancer screening via colposcopy is proposed. The significant aspects of using colposcopy images for cervical cancer screening are that it provides more focus to the patients because it is a simple and noninvasive procedure (no need to introduce instruments into the body). When compared to the other tests, the colposcopy dataset array is sparse. The automated classification of cervical cancer from colposcopy images helps mass screening for medical professionals to quickly determine whether further diagnostic checks are necessary. This paper presents the computerized system for cervical cancer prediction using colposcopy images. The critical contribution of the article is as follows:

(i) This research is aimed at developing automatic cervical cancer detection from colposcopy images using the proposed deep convolutional neural network named CYENET. Unlike previous work reported in the literature, this proposed method does not require segmentation and feature engineering stages; it can also extract the discriminative features using ensemble approaches
(ii) The transfer learning approach is used by fine-tuning the VGG19 model, which is widely used for medical image processing to predict accuracy. Besides the extensive experiment on the cancerous and noncancerous colposcopy images to effectively demonstrate the proposed CYENET (colposcopy ensemble network) and pretrained VGG model with recently proposed methods, and our proposed method achieves better accuracy as compared with the existing method in terms of classifying cervical cancer from colposcopy images
(iii) The convolutional neural network from scratch is designed to automate screening the cervical images by using an optimized architecture with an ensemble approach named CYENET (colposcopy ensemble network) deep learning architecture with a significant increase in diagnostic accuracy
(iv) Intel ODT dataset is used for experimentation. The data augmentation technique is performed on the colposcopy images to prevent the trained model's overfitting problem. This technique is an efficient strategy to learn the particular features to achieve superior accuracy
  - Another significant contribution of this paper is the use of occlusion sensitivity maps to visualize the picture characteristics of cervical cancers for classification purposes

## 3. Materials and Methods

A colposcopy image is an essential aid in early cancer diagnosis. The assessment and identification of people with irregular cytology who need further care or follow-up depend on the transition zone colposcopic examination (TZ). The title of the TZ is also an essential aspect of this study. Intra- and interobserver heterogeneity in the colposcopy perception of distinctive properties is considered to be relatively strong, but the observer heterogeneity of the TZ form and squamous column junction (SCJ) visibility evaluation and the quantitative calculation of the intra- and interobserver similarities of TZ contour tracing [37] are hardly studied. A TZ has been graded as type 1 because it is fully ectocervical (without any endocervical portion). Type 2 and Type 3 transition areas still have an endocervical component. When the latest SCJ was fully visible in TZ, it was considered a type 2. If even using external instruments, the new SCJ was not fully visible, and it was listed as type 3 [38]. It is used to assess a patient with pathological cytology, although it is not a final diagnostic examination. Variations may be made by the same colposcopies or by various colposcopies. The biggest downside of using colposcopy as a diagnostic instrument is the clinician's expertise and experience. Different experiments demonstrated good sensitivity and low accuracy in colposcopy diagnosed invasive and preinvasive cervix lesions [39].

The ensemble learning approach is employed using seven machine learning algorithms that are stacked together for automated detection for hepatocellular carcinoma [40] and using collaborative representation classification with boosting technique for classifying the hyperspectral image [41]. The flow map of the proposed automated method for detecting early cervical cancer is shown in Figure 1. The region between the original and the new SCJ is described colposcopically as the TZ [42]. The recognition of the TZ is essential information that all colposcopies require. Next, to identify the TZ as type 1, 2, or 3, you must find the new boundary between squamous and columnar epithel.  Figure 2 displays example pictures from the dataset with type 1, 2, and 3 classifications. The center image in the green is the image taken by passing the green light to improve the cervical part's visibility.

### 3.1. Deep Convolutional Neural Network Model

The CNN models have been popular in many image processing applications, including medical image analysis. Detecting cervical cancer in the colposcopy images is an obvious computer vision problem. When comparing deep learning with conventional features, the neural network, especially convolutional, is used to distinguish cases type 1, type 2, and type 3. The test is to diagnose cervical lesions using deep convolutional neural networks (moderate). The proposed VGG 19 (TL) model is fine-tuned to classify three cervical cancer classes by freezing the top layers and tested with the cervical image dataset. We proposed a CYENET architecture by incorporating the essential advantages of depth and parallel convolutional filter, to enhance the extraction of specific cervical cancer features from colposcopy images. The proposed model consists of two types of convolution layers, i.e., traditional convolution layers at the beginning of a network preceded by one single convolution filter and multiple convolution layers to extract various features from the same data. Multiple convolutional filters are used to remove the biased parts to reduce the overfitting effect. This proposed model involves three phases: (1) data preprocessing, (2) CNN model training, and (3) classification results. The CYENET model consists of 15 convolutional layers, 12 activation layers, five max pooling layers, and four cross channel normalization layers. The test data are entered into the trained model, and the output parameters are measured. The initial strata are inspired by Google net architecture, several layers for manipulating functionality, and two fully connected layers with Softmax classification layers seen in Figure 3. The network description of the CYENET model is provided in Table 2 that refers to the convolution layer and max-pooling layer, varying the filter size in the parallel convolutional block.

### 3.2. Dataset and Preprocessing

The dataset consists of 5679 colposcopy photographs obtained from the cervical screening data collection by Intel and Smartphone ODT. The data is classified by considering the transition zone visible in the diagnostic study's specific picture [36]. The dataset is preprocessed to delete all the cases' ethical details. Firstly, the data are divided into three categories through diagnostic records: type 1, type 2, and type 3. A referenced pretrained dataset identifies the area of interest (ROI) of the cervical images due to minimal professionalism with MATLAB image labeler applications' assistance. The central region in which the lesion occurs is the ROI area called the clinic's transition zone (TZ). The original picture is obtained first with annotations, marks, and ROI.

The total images are 691 cases of type 1, 3126 cases of type 2, and 1862 cases of type 3. By observing the entire dataset, it is found that the dataset is imbalanced due to its unequal distribution of images. Due to dataset imbalancing, the model maybe leads to an overfitting issue. To overcome this issue, the oversampling technique is adopted. The oversampling method is known to repeat the type 1 and type 3 images arbitrarily and equal to the number of images in type 2. The cumulative images in the data collection after the oversampling technique are 9378 images. Secondly, data enhancement methods are used to optimize the volume of training data. Using the data augmentation method, the model robustness is increased, and the overfitting problem is reduced. The input image is augmented by rotating, adjusting the brightness, cropping, and randomly increasing the dataset. After the image augmentation process, the total image size is increased to 11266. All transformed image data is eventually dimensioned to 227 × 227 for CNN to fit the model. The dataset is divided into the training data with 7498 images, validation data with 1,884, and testing data with 1,884 photos. Figures 4(a) and 4(b) display the data augmentation technique to increase the data before the input of data to train neural networks.

### 3.3. Model Parameters

In this work, the two-deep learning model is used to diagnose cervical lesions through the colposcopic images. The transfer learning VGG_19 is fine-tuned for the proposed method, and CYENET architecture developed from scratch. The standard neural network framework uses a single type of CNN filter with an input data size varying from 1 × 1 to 5 × 5. The filter convolved with the input data to produces the same input data with a discriminatory feature map. The multilayer convolutional filter design's motivation is fundamental that incorporating several convolutional filters to extracts the discrimination-based multilayer features. It extends further clusters from the same data. The three different kernel sizes are included in the training timing with 1 × 1, 3 × 3, and 5 × 5 to extract specific features. The proposed CYENET architecture and model parameters are fixed as an epoch of 50, batch size of 64, Adam optimization algorithm with a learning rate of 0.0001, and a decaying learning rate of 0.01 using piecewise technique every ten epochs. Before training, the data are shuffled at each point to bring about a normalizing effect during training. Additional discriminative features are extracted by each convolutional layer which is adding an advantage in prediction.  Figure 5(a) shows the activation map for type 1 cases extracted from the single filter from the convolutional layer 1and Figure 5(b). The activation map for type1 instances extracted from the 64 filters from the convolutional layer 1. It has been done to understand what features our CNN model is extracting for the detection of particular classes.

Mathematical equations that decide the performance of a neural network are activation functions. The functionality is attached to each neuron in the network to determine whether or not it should be triggered (“fired”), depending on input relevance with the model prediction. ReLU is a piecewise linear function that, if the input is positive, outputs directly; otherwise, it outputs zero. The ReLU activation is used due to its faster converges and avoids easy saturation. It overcomes the problem faced by logistic regression and tan hyperbolic function of an inability to output the values greater than 1. The ReLU activation function is used in all the hidden layers. It is defined as

(1) $$\begin{array}{c} f\left(x\right)=\max\left(0,x\right), \end{array}$$

where *x* is the input of the neuron. The ReLU activation function is programmed to exit the limitless activation function. The concatenation layer is used to concatenate the different features provided by the other kernel. After each concatenation layer, the local response normalization is employed to carry out the channel wise normalization of the activation function to reduce the model's overfitting problem. The local response normalization can be done in two ways: (i) within the channel and (ii) across the channel. In this proposed method, the local response normalization is carried out as cross channel normalization for pixel-wise normalization in the particular layer. It is given by equation (2).

(2) $$\begin{array}{c} x_{i}=\frac{x_{i}}{{\left(k+\left(\alpha \sum_{j}x_{j}^{2}\right)\right)}^{\beta }}. \end{array}$$

In equation two, the terms *k*, *α*, and *β*∈R are hyperparameters, and *x*_*i*_ is the input pixel value. The *A*_*x*_ pooling layer is used to minimize dimensionality after performing normalization. The max-pooling layer is used to reduce the dimension of features extracted from the convolutional layer and reduce the model's computation complexity by only keeping the channel's maximum pixel values with the specified kernel size 2 × 2. After the max-pooling layer 5, fully connected layer 1 with 128 output nodes with a drop out ratio of 0.5 is connected that follows the FC1 layer. The fully connected layer 2 with three output nodes is associated with the dropout ratio of 0.3% to reduce the overfitting problem. The softmax layer outputs each class's probabilities concerning the ground truth marks of the training and validation performance. The colposcopic images' three-class output are type 1, type 2, and type 3 to reduce the model's computation complexity instead of having 100 to 1000 nodes. The softmax activation function is indicated as

(3) $$\begin{array}{c} f_{i}\left(z\right)=\frac{e^{z_{i}}}{\sum_{g}e^{z_{g}}}. \end{array}$$

In equation (3), *f*_*i*_ is the *i*^th^ part of the class scores *f* and *z* vector, abd a vector of arbitrary real-valued scores is squashed 0 to 1 with the probability ofthe prediction rate. The categorical crossentropy function is used as the cost function to determine the error between the predicted and observed classes. The categorical crossentropy function is given in equation (4).

(4) $$\begin{array}{c} H_{p}\left(q\right)=-\overset{N}{\underset{i=1}{\sum }}y_{i}.\log\left(\left(\hat{y_{i}}\right)\right). \end{array}$$

In equation (4), $\left(\hat{y_{i}}\right)$, the *i*^th^ scalar value is in the model output, *y*_*i*_ is the corresponding target value, and *N* is the number class label (0 for type 1, 1 for type 2, and 2 for type 3). We investigated the two models CYENET and VGG 19, in the proposed process. The CYENET is developed from scratch, and the model VGG 19 is explored through the adaptation of the transfer learning process. Both the model is trained to classify the type of cervical cancer from the colposcopic images.

## 4. Results and Discussion

The experiment is implemented in MATLAB 2020b, performed on a 24 GB Quadro NVIDIA RTX 6000 workstation computer with an Intel i9 processor. Experimental data is derived from the Kaggle dataset [36]. The colposcopy cervical cancer dataset is split into 80% training, 10% validation, and 10% testing. Approximately 7498 training images and 1884 validation images are used for the training and validation process. The depth of the layer, initial learning rate, optimizer, momentum value, and L2 regularization value are calculated from the Bayesian optimization. The number of epochs is fixed as 50 for training the model. The model is trained with a multi-GPU environment, batch size of 64, and initial learning rate of 0.0001. As discussed in Section 3, CYENET and VGG 19 with fine-tuning are trained with the same image dataset with fixed parameters. The precision, sensitivity, specificity, and Cohen's kappa score are evaluated to analyze the deep learning model. The confusion matrix is also used to test the models since it deals with a multiclass classification problem. The confusion matrix is used to analyze the classification model's performance in Figure 6, the training accuracy of the proposed method VGG_19, and the CYENET model trained against the training dataset with epoch 50.

The training accuracy gradually increased concerning the epoch's number and reached the training accuracy of 97.1% for the CYENET model and 87% for the VGG_19 (TL) model. The validation plot for the proposed CYENET and the precisely tuned VGG 19 against the epoch is shown in Figure 7. The accuracy of the model is undoubtedly growing regarding the number of epochs the model is trained. After 23 epochs, the proposed CYENET model achieves the validation accuracy value of 91.3%. Simultaneously, the sophisticated VGG-19 model achieved some early oscillation in the accuracy due to the chosen learning rate of 0.0001. The VGG 19 model obtained a validation accuracy of 68.8%. The results indicate that cervical screening from colposcopic images of the CYENET model performs better than the VGG19 model due to its more robust and more straightforward architecture.

The training and validation loss curve of the proposed model CYENET and VGG 19 are shown in Figure 8. The model convergence of the proposed network is determined by the shift in the validation loss curve. Compared to the VGG 19, CYENET converges very quickly with a loss value of 0.2982, and the model VGG 19 converges to 0.9885 loss values. In comparison, the validation model of the VGG 19 is unstable, CYENET is stable, and the loss curve is smoother.

Figure 9 displays the confusion matrix for the proposed CYENET model with test data, which shows the cumulative number of images projected with accurate label correspondence to the predicted label data from the confusion matrix. The CYENET confusion matrix includes true positive (*T*_rue_ positive), false positive (*F*_alse_ positive), true negative (*T*_rue_ negative), and false negative (*F*_alse_ negative). Table 2 reports accuracy, sensitivity, specificity, positive predicted value (PPV), and negative predicted value (NPV) as our evaluation metrics. Sensitivity and specificity are the most accurate assessment metrics for classifier completeness computed from the confusion matrix in medical images.

(5) $$\begin{array}{c} \text{Accuracy}=\frac{T_{\text{rue}}\text{ Positive}+F_{\text{alse}}\text{ Negative}}{T_{\text{rue}}\text{ Positive}+T_{\text{rue}}\text{ Negative}+F_{\text{alse}}\text{ Positive}+F_{\text{alse}}\text{ Negative}}, \end{array}$$

(6) $$\begin{array}{c} \text{Sensitivity}=\frac{T_{\text{rue}}\text{ Positive}}{T_{\text{rue}}\text{ Positive}+F_{\text{alse}}\text{ Negative}}, \end{array}$$

(7) $$\begin{array}{c} \text{Specificity}=\frac{T_{\text{rue}}\text{ Negative}}{\;T_{\text{rue}}\text{ Negative}+F_{\text{alse}}\text{ Positive}}, \end{array}$$

(8) $$\begin{array}{c} \text{PPV}=\frac{T_{\text{rue}}\text{ Positive}}{T_{\text{rue}}\text{ Positiv}e+F_{\text{alse}}\text{ Positive}}, \end{array}$$

(9) $$\begin{array}{c} \text{NPV}=\frac{\;T_{\text{rue}}\text{ Negative}}{T_{\text{rue}}\text{ Negative}+F_{\text{alse}}\text{ Negative}}. \end{array}$$

Sensitivity is the percentage of people who test positive out of all those who have the disease. The proportion of people who test negative among all those who do not have the disease is the specificity of a test. The PPV is the possibility that a person will have the disease after receiving a positive test result. The NPV is the possibility that a person will not have the disease after receiving a negative test result.  Table 3 shows the test results of the proposed model tested with 1884 test images. The above experimental result CYENET model outperformed all the other models in the table trained on the colposcopic images. The DenseNet-121 and DenseNet-169 achieved lower accuracy with 72.42% and 69.79%, respectively. The model performance is influenced by the size of the dataset and also the depth of the layer. The deep architecture may decline its overall model classification performance due to the problem of interclass similarity. The Inception-Resnet-v2 model provides a lower specificity of 70.6% due to the dataset imbalance. The model is prone to image characteristics such as contrast, brightness, tone, and quality of the image capturing devices. The SVM method discussed in the performance table achieves an accuracy of 63.27% and the lowest sensitivity value of 38.46%. The model is trained on both hand-crafted features and features extracted from the CNN model. It is a time-consuming difficult task to perform in real-time even though the cost is nominal. The colponet model based on the CNN architecture provides an accuracy of 81.0% for classifying cervical cancer from the colposcopy images. The difference between the training accuracy and validation accuracy of the component model is very high. The model's training time is very high where the model is trained for 3000 epochs and provides the convergence loss of 1.12, which is very for the application of medical image processing. The proposed CYENET model is designed and trained to achieve an overall testing accuracy of 92.30% by considering all these disadvantages. The proposed model uses a different filter size to extract distinct features and works well for unexpected data. It offers a 92.40% sensitivity and a 96.20% specificity, which improves sensitivity and specificity by approximately 25% compared with Inception-Resnet-v2 in [45]. The proposed method has trouble distinguishing the false positive samples from those with fewer false positives. The CYENET model evaluates cervical epithelial features rather than morphological ones, and its false-negative epidermal features are close to true negatives. The improved sensitivity and precision indicate that positive and negative samples are predicted wisely. Since the model proposed is compared to traditional metrics such as precision, sensitivity, and specificity, sometimes, the above metrics for multiclass problems does not make sufficient to prove the model's general ability.

By taking this into consideration, the F1 score of the model is calculated by the harmonic mean of the accuracy and reminder. Still class imbalances in the dataset influence the f1 score, but Cohen's Kappa metrics are seen to have the right measure to tackle multiple class issues as well as class imbalances which the statistical standards to find the agreement between two parties. The suggested models CYENET and VGG 19 (TL), both calculated with the colposcopy images of the cervical cancer diagnosis, are measured using F1 measurements and Cohen's kappa. The F1 score of the proposed CYENET and VGG 19 (TL) is 92.0% and 44.80%, respectively, and Cohen's Kappa score of 88% and 53.5%, respectively. The proposed model CYENET is superior to the literature models and even to the proposed model VGG 19 (TL).  Figure 10 shows the graphical representation of the model discussed in Table 2.Due to the existence of several distractors such as pubic hair, intrauterine instruments, the speculum, and even human parts, the proposed method for cervical cancer screening using colposcopy can suffer. Another issue with the proposed approach if the captured images are out of focus and prediction accuracy will be reduced.

Figure 11 indicates the positive and negative expected values (PPV) of CYENET and VGG 19 models. By fixing the probability (prevalence) of infection to 0.05, the positive predicted value and negative predicted value of the CYENET model are calculated with sensitivity and specificity of 92.40% and 96.20%, respectively, for varying probabilities of infection shown in Figure 11(b), and the VGG 19 (TL) model achieves the sensitivity and specivity of 33.0% and 79.0%, respectively, for varying probability demonstrated in Figure 11(a). The incidence graph helps the medical practitioners to classify groups with a previous risk of diagnosis with cervical cancer.

The overall run time of the proposed model CYENET is 3 minutes 32 seconds, and for VGG19 5 minutes 24 seconds, the batch size of 64 is provided in Table 4. The total number of parameters for the CYENET is 8465376, and the total number of parameters for the VGG19 is 123642856. Still, the top layers are frozen to reduce the number of trainable parameters. Among the compared models, the densenet architecture proves to be having a significant training time due to its dense nature.

### 4.1. Occlusion Sensitivity Map Visualization

We used occlusion sensitivity maps [42] to determine the colposcopy images' aspects that are most appropriate for the CYENET classification decision in this experiment. Occlusion sensitivity is a simple technique for deciding which deep neural network uses image features to make a classification decision. Precisely, occlusion sensitivity measures the variation in likelihood score for a given class as a function of mask location by systematically occluding various portions of the input picture with an occluding mask (usually a grey square).  Figure 12 depicts several cervical cancer input colposcopy images with occlusion sensitivity maps superimposed on them. The occlusion sensitivity maps indicate that the colposcopy images' parts contribute more to the score for cervical cancer classes and which factors contribute less or none at all. It can be seen from the occlusion maps that CYENET was able to distinguish regions with speculum and other opacities. Compared to the Grad-CAM process, the visualization results support our argument that occlusion sensitivity maps are intuitive and interpretable.

## 5. Conclusion

A new deep learning architecture name CYENET is proposed for classifying the cervical cancer type from colposcopic images. The image dataset is balanced using the oversampling technique for improving the classification results. Two models are presented in this paper. One is using a transfer learning approach with VGG19 architecture. The other is a dedicated new model called CYENET for cervical cancer type classification using the ODT colposcopy image dataset. Both the models are evaluated using classification accuracy, sensitivity, specificity, Cohen's Kappa score, and F1-measure. The VGG19 (TL) model's sensitivity and specificity are 33% and 79%, respectively, with Cohen's Kappa score of 53.5%. The classification accuracy for VGG19 was 73.3%. Relatively satisfied results are obtained for VGG (TL). From the kappa score of the VGG19 model, we can interpret that it comes under the category of moderate classification.

Similarly, the proposed CYENET exhibited high sensitivity, specificity, and kappa scores of 92.4%, 96.2%, and 88%, respectively. The classification accuracy of the CYENET model is improved as 92.3%, which is 19% higher than the VGG19 (TL) model. Comparing the results of CYENET with previously reported results of the work, CYENET is an effective and promising prospect as a diagnosis assist tool for clinicians. The proposed method of cervical cancer classification can benefit a target population that does not need invasive intervention. The proposed CYENET has better classification efficiency and can assist medical professionals and skilled healthcare practitioners in increasing the diagnostic sensitivity and accuracy of cervical cancer detection through colposcopy screening as a result. In the future, the theoretical deep learning model will be checked for different datasets. The approach can also be enhanced by combining some advanced image processing techniques and CNN algorithms to create a diagnostic system for cervical precancerous new data.

## Figures and Tables

**Figure 1:** Flow chart of the proposed CYENET model for diagnosis of cervical cancer.

**Figure 2:** Dataset samples of type 1, type 2, and type 3 classes.

**Figure 3:** Strucutre of the proposed CYENET model.

**Figure 4:** (a) Sample input images and (b) augmented images using different techniques.

**Figure 5:** (a) Feature map of the convolutional layer with (a) 1 filter and (b) 64 filter.

**Figure 6:** Training accuracy plot for the CYENET and VGG 19 (TL) model.

**Figure 7:** Validation accuracy plot for the CYENET and VGG 19 (TL) model.

**Figure 8:** Training and validation loss curve for the CYENET and VGG_19 (TL) model.

**Figure 9:** Confusion chart of the proposed CYENET.

**Figure 10:** Performance metric comparison of systems.

**Figure 11:** PPV and NPV curve of VGG_19 (TL) (a) and CYENET (b).

**Figure 12:** Occlusion sensitivity map for test data.

**Table 1:** Summary of the related works for screening cervical cancer.

S.no	Methods	Dataset	Advantages	Disadvantages
1	Inception V3 model [1]	Herlev dataset	(i) High accuracy (ii) Good universality Low complexity	(i) The deep network needs further study to investigate cervical cells.

2	Transfer learning, pretrained DenseNet [2]	Fujian Maternal and child health hospital Kaggle	(i) More feasibility and effective	(i) Limited data

3	CNN-extreme learning machine- (ELM-) based system [6]	Herlev dataset	(i) Fast learning (ii) Easy convergence (iii) Less randomized	(i) More complexity (ii) Need more investigation

4	Gene-assistance module, voting strategy [7]	Chinese hospital and Universitario De Caracas, Venezuela	(i) More scalable and practical	(i) Limited datasets

5	Random forest and Adaboost [14]	Radiotherapy dataset	(i) Better treatment planning	(i) Need to extract features (ii) Painful treatment

6	ColpoNet [16]	Colposcopy images	(i) Better accuracy (ii) Efficient classification	(i) Need to improve accuracy by extracting relevant information

7	CNN Model [17]	Papanicolaou-stained cervical smear dataset	(i) Better sensitivity and specificity	(i) Reported 1.8% false-negative images

8	Fourier transform and machine learning methods. [18]	Microscopic images	(i) Fully automatic system (ii) Saving precious time for the microscopist	(i) The level of complexity is more

9	CNN-SVM model [21]	Herlev and one private dataset	(i) Good robustness (ii) Highest accuracy	(i) Need improvement to adjust parameter (ii) Need of hand-crafted features

10	Stacked Autoencoder [27]	UCI database	(i) High accuracy (ii) Reduced data dimension	(i) Training time is very high due to reducing the dimension

11	PSO with KNN algorithm [33]	Cervical smear images	(i) Better accuracy (ii) Good feature selection	(i) Time-consuming due to two-phase feature selection

12	Ensemble model [34]	PAP smear image	(i) For 2 class problem achieves the accuracy of 96% (ii) For 7 class problem achieves an accuracy of 78%	(i) Overall of cells are difficult to identify

13	Multimodal deep network [37]	National Cancer Institute	(i) Good correlation (ii) High accuracy (iii) Learn better complementary features	(i) More complexity in image fusion

**Table 2:** Description of network architecture of the CYENET model.

Layer No.	Layer type	Filter size	Stride	No. of filters	FC units	Input	Output
1	Convolution 1	5 × 5	2 × 2	64	—	3 × 227 × 227	64 × 112 × 112
2	Max-pool_1	3 × 3	2 × 2	—	—	64 × 112 × 112	64 × 56 × 56
3	Convolution 2	1 × 1	1 × 1	64	—	64 × 56 × 56	64 × 56 × 56
4	Convolution 3	3 × 3	1 × 1	128	—	64 × 56 × 56	128 × 56 × 56
5	Max-pool_2	3 × 3	2 × 2	—	—	128 × 56 × 56	128 × 28 × 28
6	Parallel convolution 1	1 × 1, 3 × 3, 5 × 5	1 × 1	32 ⊕ 64 ⊕ 128	—	128 × 28 × 28	224 × 28 × 28
7	Max-pool_3	3 × 3	2 × 2	—	—	224 × 28 × 28	224 × 14 × 14
8	Parallel convolution 2	1 × 1, 3 × 3, 5 × 5	1 × 1	32 ⊕ 64 ⊕ 128	—	224 × 14 × 14	224 × 14 × 14
9	Parallel convolution 3	1 × 1, 3 × 3, 5 × 5	1 × 1	32 ⊕ 64 ⊕ 128	—	224 × 14 × 14	224 × 14 × 14
10	Max-pool_4	3 × 3	2 × 2	—	—	224 × 14 × 14	224 × 7 × 7
11	Parallel convolution 4	1 × 1, 3 × 3, 5 × 5	1 × 1	32 ⊕ 64 ⊕ 128	—	224 × 7 × 7	224 × 7 × 7
12	Max-pool_5	5 × 5	1 × 1	—	—	224 × 7 × 7	224 × 2 × 2
13	Fully connected 1	—	—	—	512		
14	Fully connected 2	—	—	—	3		

**Table 3:** Comparative experiment results of proposed architecture with different models.

Model name	Accuracy (%)	Sensitivity (%)	Specificity (%)	PPV (%)	NPV (%)	Ref
DenseNet-121	72.42	59.86	76.83	48.39	84.52	[43]
DenseNet-169	69.79	65.00	71.48	44.84	85.31	[43]
Colponet	81.0	—	—	—	—	[16]
SVM	63.27	38.46	71.85	32.43	76.87	[44]
Inception-Resnet-v2	69.3	66.70	70.6	47.20	84.00	[45]
CYENET	92.30	92.40	96.20	92.00	95.00	Present study
VGG19 (TL)	73.30	33.00	79.00	70.00	88.00	Present study

**Table 4:** Comparative results of proposed architecture with several parameters and run time.

Model name	Number of parameters	Run time (per epoch)
DenseNet-121 [43]	7978856	21 min 10 s
DenseNet-169 [43]	28681000	24 min 59 s
Colponet [16]	6977000	16 min 27 s
Inception-Resnet-v2 [45]	55843161	15 min 36 s
CYENET	8465376	3 min 32 s
VGG19 (TL)	123642856	5 min 24 s

## Data Availability

The data used to support the findings of this study are included within the article.
